The article "Edge AI-Based Automated Detection and Classification of Road Anomalies in VANET Using Deep Learning" was published in 2021. Journal: Comput Intell Neurosci.

# Edge AI-Based Automated Detection and Classification of Road Anomalies in VANET Using Deep Learning

**DOI:** 10.1155/2021/6262194

**Published:** 2021-09-29

**Authors:** Rozi Bibi, Yousaf Saeed, Asim Zeb, Taher M. Ghazal, Taj Rahman, Raed A. Said, Sagheer Abbas, Munir Ahmad, Muhammad Adnan Khan

**Affiliations:** ^1^Department of Information Technology, The University of Haripur, Haripur, Pakistan; ^2^Department of Computer Science, Abbottabad University of Science and Technology, Havelian, Pakistan; ^3^Center for Cyber Security, Faculty of Information Science and Technology, Universiti Kebangsaan Malaysia (UKM), 43600 Bangi, Selangor, Malaysia; ^4^School of Information Technology, Skyline University College, University City Sharjah, 1797 Sharjah, UAE; ^5^Department of Physical & Numerical Science, Qurtuba University of Science & Information Technology, Peshawar 25000, Pakistan; ^6^Canadian University Dubai, Dubai, UAE; ^7^School of Computer Science, National College of Business Administration and Economics, Lahore 54000, Pakistan; ^8^Pattern Recognition and Machine Learning Lab, Department of Software, Gachon University, Seongnam 13120, Republic of Korea

## Abstract

Road surface defects are crucial problems for safe and smooth traffic flow. Due to climate changes, low quality of construction material, large flow of traffic, and heavy vehicles, road surface anomalies are increasing rapidly. Detection and repairing of these defects are necessary for the safety of drivers, passengers, and vehicles from mechanical faults. In this modern era, autonomous vehicles are an active research area that controls itself with the help of in-vehicle sensors without human commands, especially after the emergence of deep learning (DNN) techniques. A combination of sensors and DNN techniques can be useful for unmanned vehicles for the perception of their surroundings for the detection of tracks and obstacles for smooth traveling based on the deployment of artificial intelligence in vehicles. One of the biggest challenges for autonomous vehicles is to avoid the critical road defects that may lead to dangerous situations. To solve the accident issues and share emergency information, the Intelligent Transportation System (ITS) introduced the concept of vehicular network termed as vehicular ad hoc network (VANET) for achieving security and safety in a traffic flow. A novel mechanism is proposed for the automatic detection of road anomalies by autonomous vehicles and providing road information to upcoming vehicles based on Edge AI and VANET. Road images captured via camera and deployment of the trained model for road anomaly detection in a vehicle could help to reduce the accident rate and risk of hazards on poor road conditions. The techniques Residual Convolutional Neural Network (ResNet-18) and Visual Geometry Group (VGG-11) are applied for the automatic detection and classification of the road with anomalies such as a pothole, bump, crack, and plain roads without anomalies using the dataset from different online sources. The results show that the applied models performed well than other techniques used for road anomalies identification.

The article "Edge AI-Based Automated Detection and Classification of Road Anomalies in VANET Using Deep Learning" was published in 2021. Journal: Comput Intell Neurosci.

## 1. Introduction

In our daily life, road conditions play an important role. Road pavement irregularities can lead to mechanical failure of vehicles and may cause accidents. Poor road conditions also affect the comfort of drivers and passengers and increase stress levels [1]. According to World Health Organization (WHO) 2018 report survey, every year 1.35 million people lose their lives in road accidents. The rate of road mortality in low- and middle-income countries having 60% of the world's vehicles is more than 90%. The leading cause of death in the world population aged in the range of 5–29 years is road traffic injuries (WHO, 2018) [2]. The rate of deaths in road traffic injuries varies in numbers for different Asian countries from the year 2009 to 2018. The number of deaths in fourteen Asian countries such as Afghanistan, Bangladesh, China, India, Iran, Japan, Kazakhstan, Kyrgyzstan, Malaysia, Pakistan, Philippines, Sri Lanka, Turkey, and Vietnam is compared by using data from World Health Organization reports published on global road safety in 2009, 2013, 2015, and 2018 [2–5], as shown in Figure 1.

Road accidents due to adverse conditions of the road and over speed may lead to life-threatening injuries such as head trauma, damage to the brain, injury to the neck or back, fractured bones, injuries to the eyes, and other internal injuries. Damaged roads also increase the fuel consumption in vehicles. To minimize accidents rate and mechanical failures in vehicles, road systems need to be regularly inspected in the field of highway building and road safety to recognize threats of damage and possible risks [6]. Terrible road conditions such as rough roads, potholes, cracks, manholes, speed bumps, ditches, and surface height imbalance are major sources of vehicle crashes and high death rates. The concrete material quality, large rate of traffic flow, heavy vehicles, and climate changes such as snowfall and heavy rains are affecting road surfaces, and as a result, road anomalies are increasing day by day [7]. Road surface anomalies are becoming an increasingly important issue for roads around the world, such as potholes and cracks.

To prevent a vehicle from damage that occurs due to over speed, the early detection of speed bumps is necessary. Moreover, the detection of anomalous road surfaces and any other hurdle causing the problem in the smooth traffic flow is vital in the Intelligent Transportation System (ITS) by using in-vehicle sensors and their measurements for reducing possible harm to the vehicles and humans [8, 9]. The vehicular ad hoc network (VANET) is a special case of a wireless multihop network introduced by ITS [10]. Each vehicle in a network receives data that is transmitted by other vehicles and also shares their data with other devices within a network. After accumulating all such data, the nodes would then work to extract useful information from the data, and then, the information is sent back to other devices. VANET communication is categorized into Vehicle-to-Vehicle (V2V), Vehicle-to-Infrastructure (V2I), and Infrastructure-to-Infrastructure (I2I) communication. Furthermore, in a critical situation, the exchange of useful pieces of information to other vehicles in a network is vital for safety purposes. Dedicated Short-Range Communications (DSRC) are benchmarks for vehicular remote communication. A DSRC is a free and authorized range conveyed by the United States Federal Communications Commission (FCC) to support communication inside the range of 300 m to 1 km [11].

The article "Edge AI-Based Automated Detection and Classification of Road Anomalies in VANET Using Deep Learning" was published in 2021. Journal: Comput Intell Neurosci.

Today, autonomous vehicles (AVs) are an active research area with advantages for disabled people, old people, and less energy consumption especially after the emergence of deep learning techniques [12]. Deep Neural Networks (DNNs) have become leading technologies in many areas due to their astonishing features, allowing vehicles to interpret their driving environment and to take actions accordingly [13]. Artificial Intelligence strategies will provide autonomous vehicles with promising solutions for the perception of the environment and with sufficient decision-making for smooth navigation [14]. Deep learning also supports traditional, humanly designed computer vision approaches, particularly in the area of visual data processing. End-to-end autonomous driving control based on learning has the advantage that the device design is streamlined because CNN learns without clear knowledge of the surrounding environment and motion planning automatically and is reliable. However, end-to-end CNN-based learning has a problem where the basis of the importance of output control is not understood. Research is being carried out on an approach based on judgment to resolve this issue, such as turning the steering wheel to the left or right and stepping on brakes that can be understood by people [15]. A well-trained deep learning model can be deployed on cloud or edge devices for inference [16]. The deployment of a trained deep learning model in the autonomous ground vehicle for road anomalies detection will be very useful for obtaining efficiency in the autonomous field. Using a combination of sensors and DNN techniques, unmanned vehicles can perceive their surroundings for the detection of tracks and obstacles for smooth traveling. The controller takes images and forecasts details to visual navigation devices to enable autonomous vehicles for the perception of surroundings. However, to bring the concept of an autonomous vehicle to life many major manufacturers, including Tesla, GM, Ford, BMW, and Waymo/Google are involved in the construction and testing of various types of autonomous vehicles [17]. These modern autonomous vehicles are equipped with many sensors such as an accelerator, a Global Positioning System (GPS), fuel sensor, pressure sensor, ultrasonic sensor, radar, camera, lidar, rain sensor, thermal sensor, and many other sensors for automatic checking of oil, temperature, pressure and coolant level, etc. Each sensor performs a specific function and accomplishes relevant tasks for a steady flow of traffic. An autonomous vehicle's working architecture is composed of four major layers i.e., sensor, perception, planning, and control layer incorporating an intelligent system that monitors the environment, makes decisions, and takes action based on these decisions [13].

The article "Edge AI-Based Automated Detection and Classification of Road Anomalies in VANET Using Deep Learning" was published in 2021. Journal: Comput Intell Neurosci.

However, the biggest challenge for autonomous vehicles is to avoid the critical road anomalies that lead to dangerous accidents and financial crises for manufacturers [18]. To prevent a collision with road anomalies, an autonomous vehicle needs not only to detect anomalies but also to find an alternative safe path and guide itself in real time to a secure and productive direction [19]. For the detection and classification of road anomalies for the safe and smooth navigation of vehicles, various studies have been conducted by the research community. These studies present input data from various sensors and using different machine and deep learning algorithms for the identification of road anomalies such as potholes, cracks, bumps, manholes, and any other static objects that are a source of road accidents and mechanical failure in vehicles. Various machine learning, image processing, and deep learning approaches have been used by researchers for this purpose based on vision sensors and vibration sensors, 3D laser scanner, and 2D images [20]. The related study is discussed in the context of vision-based methods and vibration-based methods used for the detection of road anomalies.

Vision-based methods are cost-effective and able to provide a fast real-time prediction of road anomalies for solving road anomaly automatic detection challenges in vehicles. However, these methods are affected by weather and lighting conditions in the real world. In [21], satellite images and road maps are used for the detection of road anomalies. The UNet is used for binary classification of road and nonroad regions, and a modified form of DeepLab e.g. deeplabv3+ is used for multiclassification of three types of road surfaces such as pavement, concrete, and gravel. The authors in [22] prefer the deep learning approaches for black box images. The proposed model is based on two CNN models for road features extraction and crack detection. The CNN1 model is used to reduce the region of the crack detection area, and the CNN2 model classifies the images into three classes, namely, cracks, intact area, and road marking with 81.79% *F*-measures, 90.81% precision, and 74.4% recall. In [23], the detection of potholes from collected images by authors is done by using Single-Frame Stereo Vision-Based Method (SV1), Multiframe Fusion-Based Method (SV2), Mask R-CNN (LM1), and YOLOv2 (LM2). The rate of precision and recall for SV1 is 45.8% and 45.8%, for SV2 is 67.4% and 51.2%, and for LM1 is 89.8% and 92.8%, while the LM2 model is capable of detecting potholes in real time. In [24], the real-time detection of five classes of road damages from images i.e., longitudinal crack, horizontal crack, alligator damage, pothole-related crack, and line blurring is accomplished by using a single-shot multibox detector (SSD) and faster region-based convolutional neural networks (R-CNN) with Inception V2 and ResNet. The results show that the achieved accuracy rate of 0.5306 for Inception ResNet V2 is better than other approaches. In [25], the fully convolutional neural network (FCN) with VGGNet as a backbone is used for the detection of the crack based on semantic segmentation of images. The experimental result shows that the proposed method achieves performances of 91.3%, 94.1%, 92.1%, and 92.8% for the precision, recall, *F*_1_-score, and SA, respectively.

The article "Edge AI-Based Automated Detection and Classification of Road Anomalies in VANET Using Deep Learning" was published in 2021. Journal: Comput Intell Neurosci.

Deva Priya et al. proposed a methodology based on image processing and morphological techniques for a private dataset in [26] for the detection of five kinds of road speed bumps that vary in width, height, and color with an accuracy of 84.5%. In [27], the binary transformation and morphological operations are used for reducing noise and extraction of features from private images dataset, and the decision tree method is adopted for the classification of superficial cracks, crocodile cracks, linear cracks, transverse cracks, and road without cracks. The experimental results prove the efficiency of the proposed methodology through good results and show that this approach can be utilized for solving a real-world problem promptly. Furthermore, low-pass Gaussian filter and median filtering image processing techniques have been utilized in [28] for the detection of five different categories of speed bumps based on color in images. The proposed method performs successfully for four categories of speed bumps with an accuracy of 90% and below average for the fifth category of the speed bump. Furthermore, Yolov3, SSD, HOG, and Faster-RCNN deep learning models are used for the detection of potholes with an accuracy of 82%, 80%, 27%, and 74%, respectively, in [29]. Gopalakrishnan et al. in [30] used a pretrained deep convolutional neural network VGGNet-16 and multiple classifiers i.e., Single-Layer Neural Network (NN), Random Forest (RF), Extremely Randomized Trees (ERT), Support Vector Machine (SVM), and Logistic Regression (LR) for the binary classification of cracks for their dataset. In the presented solution, the image vector produced by VGGNet-16 is further used as input to classifiers. The experimental results show that the performance of NN with transfer learning is higher than other approaches. The crack detection accuracy percentage for NN, RF, ERT, SVM, and LR is 90%, 86%, 87%, 87%, and 88%, respectively. Dalia et al., in [31], worked for potholes and cracks detection based on morphological algorithms; the Gaussian low-pass filter is used for noise reduction in images, and Otsu's algorithm is used for obtaining cell pixels' values based on threshold values, and to get the connected pixels only, morphological algorithms-based skeletonization technique is used.

In [32], Li et al. used FC-DenseNets for crack detection with a recall of 96.63% on publicly available CFD and AigleRN datasets. In [33], CNN and SVM classifiers are used for detection and binary classification of potholes' images collected from multiple sources and attained accuracy of 99.80% for CNN and 88.20% for SVM. Vosco Pereira et al., in [34], applied Tensorflow API and achieved a precision rate of 97.46% for the real-time detection of road bumps from their dataset that is also available publicly. In [35], Yolov2 is used by Bhanu Prakash et al. for potholes detection using a publicly available potholes' dataset. The experimental results show that the applied method worked successfully with a precision of 95.55%. Moreover, deep learning classifiers' CNN-based ResNet models are used for pothole classification based on thermal images in [36] with an accuracy of 97.08%. In [37], potholes are detected via CNN obtaining an accuracy of 95%. In [38], for detection of cracks, the authors used a machine learning approach i.e., CrackForest (One-Class SVM) on the CFD dataset and attained 96.73% precision. In [39], CNN has applied on their own images dataset for crack detection. The proposed CNN model worked successfully by attaining 92.51% recall. In [40], CNN is proposed for the detection of speed bumps and the authors used an additional image processing technique for the case in which CNN fails to detect speed bumps. Suong et al. used Yolov2 for potholes detection by collecting potholes images from Google in [41] and achieved 82.43% precision and 83.72% recall. In [42], MobileNetV2, EfficientNetB0, DenseNet201, and InceptionV3 deep learning models are used for the detection of concrete cracks from image datasets from multiple sources. The proposed models attained successful experimental results with accuracy of 97.82%, 99.11%, 99.32%, and 98.89%, respectively. In [43], an improved version of the VGG16 network for the detection of crack is presented, and the authors prepared their dataset, named CCD1500, for training the model, whereas the CFD, DeepCrack, and CrackTree200 datasets are used as test data. The experimental results indicate that the proposed model gained successful detection results with a recall of 90.30% for CFD, 96.60% for DeepCrack, and 89.10% for the CrackTree200 dataset.

The article "Edge AI-Based Automated Detection and Classification of Road Anomalies in VANET Using Deep Learning" was published in 2021. Journal: Comput Intell Neurosci.

In [44], the fully convolutional network based on pretrained deep learning models VGG16, Inception v3, and ResNet is applied on concrete crack images with accuracy performance of 99.99% for VGG16, 99.90% for Inception v3, and 97.50% for the ResNet model. Fan et al., in [45], classified the crack using CNN model. Moreover, the threshold techniques are used for the segmentation of images with achieving 99.92% precision results for classification and 98.70% for segmentation of cracks. For real-time detection of crack defects, Akarsu et al., in [46], used a morphological image processing approach for features extraction and decision tree for crack classification. From implementation details, it can be depicted that the method works successfully for the real-time detection of defects. In [47], canny edge detector technique is applied to real-world images for the detection of potholes. The precision and recall for pothole detection using the canny edge detector reach up to 81.80% and 74.4%, respectively. In [48], the pothole detection from images is based on three steps. Firstly, the dark regions of potholes are detected and extracted by applying a histogram and the closing operation of a morphology filter. Secondly, the candidate features of potholes such as compactness and size are extracted. Finally, the pothole is detected based on candidate features. The proposed approach attained 73.50% accuracy, 80% precision, and 73.30% recall. Young-Ro et al., in [20], proposed an IoT-based alert system for pothole detection using images. The collected images are converted into the binary form; then, a matching value is searched in the database for detection of potholes. In [49], image segmentation methodologies for potholes detection such as thresholding, edge detection, *K*-means clustering, and fuzzy *C*-means clustering are proposed and applied on images collected from Google by authors. The average accuracy segmentation performance for thresholding technique is 80.60%, for edge detection is 90.19%, for *K*-means clustering is 82.47%, and for fuzzy *C*-means clustering is 82.46%. However, the computation time for *K*-means clustering is less than other approaches and can be preferable for fast computation. In [50], the CNN model is used for the detection of crack with an accuracy achievement of 70.7%. In [51], the Inception V2 deep learning model is used for pothole images from the video. In [52], the authors have chosen the modified version of AlexNet, i.e., SqueezeNet, which is faster in speed and smaller in size than AlexNet. The SqueezeNet is applied on GAPs and ICIP datasets for detection of cracks and potholes attaining accuracy of 99.89% for the GAPs' dataset and 92.37% for the ICIP dataset. In [53], potholes are detected in asphalt pavement images using supervised learning. The features are extracted using HOG and Naive Bayes classifier to localize the pothole over the region. The obtained results are 90.0%, 86.50%, and 94.10% for accuracy, precision, and recall.

The article "Edge AI-Based Automated Detection and Classification of Road Anomalies in VANET Using Deep Learning" was published in 2021. Journal: Comput Intell Neurosci.

Vibration-based methods are suitable for real-time detection of road anomalies with consumption of less storage. These methods are highly susceptible to error due to sensitivity to frequency noise and signals from other sensors working in the vehicle. Moreover, the vibration effect produced by any other obstacle on road similar to road anomalies can be detected as road anomalies. Several efforts have been made by researchers for the detection of road anomalies based on the vibration method. In [54], the authors used a gyroscope and accelerometer for speed bump detection and upload resultant values on a cloud server for smooth navigation. The gyroscope is used for measuring gravity changes and the accelerometer for linear velocity. Data is collected through mobile phone sensors, and a Butterworth filter is used for reducing noise. *Z*-axis readings of the accelerometer and *X*-axis readings of the gyroscope are used for the extraction of features based on standard deviation, mean, and min-max value, and speed bumps and smooth roads are classified by applying Support Vector Machine (SVM) using RBF, MLP, and polynomial kernels that achieved an accuracy rate of 75.76%, 66.67%, and 87.88%, respectively. In [55], the detection method for speed bumps on road by You Member et al. involves sensing the environment using the mobile phone gravity sensor and GPS sensor. The collected data for speed bumps detection is passed to a cloud unit composed of API, database, and data-mining layers for generating accurate data, storage and applying the *K*-mean clustering technique, respectively, whereas Bluetooth is used for communication between the microcontroller and vehicle for controlling speed. In [56], the authors address the problems associated with roads without infrastructure by utilizing accelerometer and GPS sensors of mobile phones for sensing the road obstacles and classify the road obstacles into two categories. The first category contains actionable obstacles such as potholes, utility patches, drains, catch basins, sunk casting, animals, moving humans, construction material, and speed bumps that are caused by natural factors, whereas the other category contains nonactionable obstacles including train tracks and flat casting that have the least dangerous effects. Road features i.e., latitudinal and longitudinal parameters, speed, and accelerometer coordinates are recorded through mobile sensors, and the beta-signature filter is applied for classification.

The article "Edge AI-Based Automated Detection and Classification of Road Anomalies in VANET Using Deep Learning" was published in 2021. Journal: Comput Intell Neurosci.

Song et al., in [57], proposed an effective strategy for pothole detection by utilizing a gyroscope and accelerometer. The convolutional neural network (CNN) model Inspection V3 is used for the classification of the three categories of road anomalies i.e., normal, pothole, and bumps, and the accuracy of classification is approaching 100%. Furthermore, roads classified into paved and unpaved roads, and the work is proposed in [58] using an android application for obtaining data from mobile phone accelerometer, gyroscope, GPS, and compass. Support Vector Machine (SVM), Hidden Markup Model (HMM), and ResNet models are used for the classification of paved and unpaved roads, whereas for the detection of the road anomaly and smooth road, the KNN strategy is utilized based on Dynamic Time Warping (DTW) based on Euclidean distance approach for paved roads. The accuracy obtained for the classification of paved and unpaved roads using SVM, HMM, and ResNet is 96%, 85%, and 97%, respectively. In [59], the road monitoring system based on the Internet of Things (IoT-RMS) for potholes is proposed by the authors. An accelerometer, ultrasonic sensor, and global positioning system (GPS) sensors are used for data collection. Cloud server and Honey Bee Optimization (HBO) algorithm are adopted for pothole detection.

The article "Edge AI-Based Automated Detection and Classification of Road Anomalies in VANET Using Deep Learning" was published in 2021. Journal: Comput Intell Neurosci.

The authors in [60] applied principal component analysis (PCA) technique-based detection of the anomalies belonging to four classes i.e., long bumps, short bumps, manhole, no anomaly, and others are proposed by authors using speed, GPS coordinates, and accelerometer data. The web-based application is designed for anomaly detection. The accuracy for anomaly detection in a laboratory environment is 94.69%, and in a real-world scenario, the accuracy is 82.51%. Varona et al., in [61], proposed a model based on deep learning for automatic detection of vehicle stability on defective roads. The data about various road surfaces such as concrete panels, cobblestones, asphalt, and dirt roads are collected through smartphones' accelerometer and GPS sensors. Convolutional neural network (CNN), long short-term memory neural network (LSTM), and reservoir computing (RC) are stable classifiers for road annomilies detection. The experimental results show that the CNN model has better performance than other approaches and achieved an accuracy rate of 85% for road surface classification and 93% for stability events. In [62], the proposed model includes data collection from mobile phone sensors i.e., accelerometer and GPS. To remove the noisy data, the Butterworth filter is used and the Gaussian background model is utilized with improvements according to the need for abnormal road recognition, whereas the abnormal road surfaces are classified using the KNN algorithm for the detection of potholes and speed bumps on roads with an accuracy rate of 94.12% and 96.03%, respectively. In [63], the authors highlighted the problems in various techniques that have been used for anomaly detection. The proposed methodology involves the collection of data through the accelerometer of the smartphone; then, anomalies are located by using threshold detection and sliding window technique. Moreover, for the classification of a pothole, metal bumps, and speed bumps, the Dynamic Time Warping technique based on KNN is used.

Several machine learning and deep learning techniques have been applied for different types of road anomalies detection. However, in terms of performance, improvement is needed. One of the major causes for high road accidents rate and deaths are road surface damages due to natural disasters which is common throughout the world specifically in Asian and underdeveloped countries. With the emergence of AI-powered devices and the benefits of an intelligent transportation system, these road hazards can be minimized. In the proposed system, with the help of powerful computational capabilities in smart devices based on artificial intelligence and the benefits of vehicular ad hoc networks, road surface conditions can be communicated within a network of vehicles. The proposed research work is helpful for the society by considering an intelligent mechanism in a vehicle for early detection of road conditions and resolving problems of road accidents, deaths, and vehicles damage.

The article "Edge AI-Based Automated Detection and Classification of Road Anomalies in VANET Using Deep Learning" was published in 2021. Journal: Comput Intell Neurosci.

The present study is based on vision-based methods for automatic detection and classification of road anomalies images into four classes i.e., potholes, road bumps, cracks, and plain road (no anomaly) using ResNet-18 and VGG-11 deep learning models. To solve the problems related to road anomalies on the rough road surface for smooth traffic flow and reducing hazards, an Edge AI-based framework for automatic identification of pothole, crack, speed bump, and plain road (no anomaly) is proposed for an autonomous vehicle in this study, as shown in Figure 2. In the proposed framework, the VANET environment is used for maintaining the safety of vehicles through message broadcasts related to road conditions to incoming vehicles. The road anomalies concerning its type(s) are recognized by using any trained deep learning model deployed in a vehicle embedded powerful processor and further can be used for path planning and avoidance mechanism in autonomous vehicles.

The rest of the paper is organized as follows. In Section 2, proposed methodology with a description of the dataset and proposed deep learning models are explained. Results are described and compared in Section 3, and the conducted study is concluded in Section 4 with possible future research directions.

## 2. Materials and Methods

In this section, we present the proposed methodology that involves a description of the dataset used for the study, preprocessing of the data for removing noisy and repeated data, and data augmentation technique for increasing the quantity of the dataset, as shown in Figure 3. Furthermore, the deep learning models used for the classification of road anomalies are described at the end of Section 2.

### 2.1. Data Analysis

The dataset is collected from different online sources. Pothole dataset is collected from [64] which consists of images of the dry, water-filled, and dusty potholes of various shapes captured in clear and low light weather conditions. For bump detection, the publicly available dataset from [65] is utilized that has marked as well as unmarked road bumps images, whereas the CFD and Aigle crack datasets which consist of low severity cracks having width 0.1 mm–0.3 mm are used for crack detection [38]. In the case of no anomaly, the plain road dataset is collected from [66]. The collected data is preprocessed before passing to training models.

The article "Edge AI-Based Automated Detection and Classification of Road Anomalies in VANET Using Deep Learning" was published in 2021. Journal: Comput Intell Neurosci.

### 2.2. Preprocessing

The preprocessing stage involves cleaning duplicated data, removing unnecessary parts from images, and augmentation techniques. The deep learning model needs a large dataset for training and enhancing performance. To improve the performance of deep learning models with a small dataset, data augmentation plays a vital role [67]. To reduce overfitting in deep learning models, different data augmentation techniques such as zooming, cropping, horizontal shift, and rotation are applied to our dataset to increase the dataset for deep learning models. The number of images in the original dataset and dataset after augmentation related to different road anomalies is shown in Table 1.

### 2.3. Deep Learning Models

After preprocessing, the dataset is passed to CNN models for training procedure. In this research, CNNs are used instead of using conventional machine learning techniques that are provided with hand-crafted characteristics to learn and take time and effort. CNN's have the power to learn from raw data automatically. Different CNN models such as AlexNEt [68], ResNet [69], DenseNet [70], and VggNet [71] have been utilized by the authors for the automatic detection and classification of images in different fields. The transfer learning approach for deep learning models saves time and computation resources [72]. In the presented work, two powerful state-of-the-art architectures of CNN based on transfer learning are used for the classification and identification task of road anomalies detection. On the ImageNet Large-Scale Visual Recognition Challenge (ILSVRC) dataset, these models are successfully trained. Furthermore, another common object localization method is gradient-weighted class activation mapping (Grad-CAM) [15], which uses gradient values determined during the backpropagation process to produce an attention map for locating a particular object in the image.

#### 2.3.1. ResNet-18

One of the most common convolution neural networks (CNN) is a deep residual network (ResNet) which was proposed by He et al. in 2015 that performs best in the classification of the image for the ImageNet database [73]. ResNet-18 is a pretrained deep learning model with 18 layers. It is consists of 16 convolution layers, 2 down-sampling layers, and some fully connected layers (FC). The input image size of ResNet is 224 × 224, and in addition to the first convolution layer, the convolution kernel size is 7 × 7, and in the other layers, it is 3 × 3. After average pooling the feature map of the last convolution layer, an eigenvector is obtained by full connection; then, the classification probability is obtained by normalization with Softmax. The general architecture of ResNet-18 is shown in Figure 4 for road anomalies automatic detection and classification into four classes.

The article "Edge AI-Based Automated Detection and Classification of Road Anomalies in VANET Using Deep Learning" was published in 2021. Journal: Comput Intell Neurosci.

#### 2.3.2. VGG-11

VGGNet is a very deep convolutional network and was introduced by Simonyan and Zisserman in 2014 [74]. It is the most widely used pretraining convolution architecture for the ImageNet dataset. The biggest success of this network is that the depth of the network is high, which is important to ensure good performance. The VGGNet version VGG-11 is comprised of a total of 11 layers. It consists of 8 convolutional layers, two fully connected layers, and an output layer with Softmax. Each layer is convolved with 3 × 3 convolution with a feature map of sizes 64, 128, 256, and 512, respectively. The general architecture of VGG-11 for road anomalies automatic detection and classification into four classes is shown in Figure 5.

## 3. Results and Discussion

This section describes the experimental input parameters for training pretrained deep learning models and comparison of proposed models with the previous approaches used for different types of road anomalies. The experimental results are carried out on Google Colab [75] and implemented in Python language using the fastai library [76]. The input parameters for training deep learning models are listed in Table 2.

The confusion matrix is used for performance analysis. True positive (TP) represents the true positive rate and points out the positive class determined as positive. False positive (FP) is a false positive rate that represents the negative class determined as positive, whereas the false negative (FN) refers to a positive class determined as negative, and true negative (TN) is the true negative rate that points out the negative class determined as negative [77]. The performance of proposed deep learning models is evaluated based on precision, recall, accuracy, and *F*_1_-score.

Precision is also termed as a positive predicted value, and it can be calculated by using the following equation:

(1) $$\begin{array}{c} \text{Precision}\left(\text{Prc}\right)=\frac{\text{TP}}{\text{TP}+\text{FP}}. \end{array}$$

The number of positive class predictions made from all positive examples in the dataset is quantified by the recall. The mathematical expression for the recall is represented in the following equation:

(2) $$\begin{array}{c} \text{Recall}\left(\text{Rec}\right)=\frac{\text{TP}}{\text{TP}+\text{FN}}. \end{array}$$

The proportion of a total number of correct predictions in a confusion matrix for a particular class is termed accuracy and can be estimated through the following equation:

(3) $$\begin{array}{c} \text{Accuracy}\left(\text{Acc}\right)=\frac{\text{TP}+\text{TN}}{\text{TP}+\text{TN}+\text{FN}+\text{FP}}. \end{array}$$

*F*_1_-score provides a single score that balances both the concerns of recall and precision in one number. The mathematical formula for the *F*_1_-score is represented in the following equation:

(4) $$\begin{array}{c} F_{1}-\text{Score}\left(\text{Fs}\right)=2*\frac{\text{Prc}*\text{Rec}}{\text{Prc}+\text{Rec}}. \end{array}$$

Moreover, the learning curve is a plot of the performance of model learning. In machine learning, learning curves are a commonly used diagnostic method for algorithms that learn incrementally from a training dataset. After each update during training and plots of the measured performance can be generated, the model can be tested on the training dataset and a holdout validation dataset [78]. The learning curve for the deep learning model ResNet-18 is shown in Figure 6. Figure 6 indicates that the training and validation loss for ResNet-18 are nearly approaching 0 which means that the proposed model trained well.

The article "Edge AI-Based Automated Detection and Classification of Road Anomalies in VANET Using Deep Learning" was published in 2021. Journal: Comput Intell Neurosci.

The confusion matrix for ResNet-18 obtained for the classification of road anomalies is shown in Figure 7. The diagonal values in the confusion matrix represent the instances of a particular class that are predicted correctly. It can be depicted from Figure 7 that the efficiency of the proposed models is high for making predictions of road anomalies. The truly predicted value (TP) for road anomaly type bump is 334, for crack is 327, for pothole is 373, and for no anomaly case is 322.

The evaluation parametric results for road anomaly types are presented in Table 3. It can be exhibited from Table 3 that the prediction precision of ResNet-18 for bump is 100%, recall is 99.70%, accuracy is 99.92%, and *F*_1_-score is 99.84%. In the case of crack, the prediction precision, recall, accuracy, and *F*_1_-score of ResNet-18 is 100%. Furthermore, the predicted precision, recall, accuracy, and *F*_1_-score of ResNet-18 for the no anomaly case are 99.38%, 100%, 99.85%, and 99.68%, respectively. In the case of the pothole, the prediction precision of ResNet-18 is 100%, recall is 99.73%, accuracy is 99.92%, and *F*_1_-score is 99.86%.

Moreover, the learning curve for the deep learning model VGG-11 is shown in Figure 8. Figure 8 shows that the training and validation loss for VGG-11 both are decreasing gradually, and at the end of training, these are nearly approaching 0.Whereas Figure 9 represents the confusion matrix for VGG-11. The truly predicted value (TP) for road anomaly type bump is 300, for crack is 342, for pothole is 349, and for no anomaly case is 365.

For VGG-11, the prediction precision for bump, no anomaly, and pothole is 100%. The predicted recall of VGG-11 for bump, crack, and no anomaly cases are 100%. Moreover, the predicted accuracy and *F*_1_-score for bump and no anomaly cases is also 100%. For crack, the prediction precision of VGG-11 is 99.41%, accuracy is 99.85%, and *F*_1_-score is 99.70%, whereas, in the case of pothole, the prediction recall, accuracy, and *F*_1_-score of VGG-11 are 99.43%, 99.85%, and 99.71% as presented in Table 4.

The article "Edge AI-Based Automated Detection and Classification of Road Anomalies in VANET Using Deep Learning" was published in 2021. Journal: Comput Intell Neurosci.

The performance of both models is compared based on average accuracy achieved for the classification of road anomalies as represented graphically in Figure 10.

The performance of the proposed models is compared with the deep learning, machine learning, and image processing techniques that are previously implemented by researchers in Table 5. The results for potholes detection are compared with the techniques CNN, SVM, Yolov2, Naive Bayes, *K*-means clustering, fuzzy *C*-means clustering, and morphological algorithm used in [33, 35, 48, 49] and [53], respectively, as shown in Figure 11.

In the case of bump, the performance of proposed models is compared with proposed methodologies such as TensorFlow API and image filtering morphological algorithm in [26, 28, 34] as presented in Figure 12.

Furthermore, the results of the techniques used by authors in [30, 41] that are Neural Network (NN), Random Forest (RF), ERT, SVM, LR, MobileNetV2, EfficientNetB0, DenseNet201, and InceptionV3 are compared with results of ResNet-18 and VGG-11 for crack detection, as described in Figure 13.

## 4. Conclusions and Future Work

In this study, an Edge AI-based framework is suggested for the road anomalies detection for an autonomous vehicle. In this proposed mechanism, trained deep learning model deployment at the vehicle level is used for the prediction of the road anomaly class. To solve the accident issues and sharing emergency information, the Intelligent Transportation System (ITS) introduced the concept of the vehicular network termed as vehicular ad hoc network (VANET) for achieving security and safety in a traffic flow. Road images captured via camera and deployment of the trained model for road anomaly detection in a vehicle could help reduce the accident rate and risk of hazards on poor road conditions. For the automatic detection and classification of the road with anomalies such as a pothole, bump, crack, and plain road without anomalies, the pretrained deep learning models ResNet-18 and VGG-11 are used. The dataset is collected from different online sources. An open-source Google Colab and fastai library are used for obtaining results. The experiment results demonstrated that the suggested models supersede the other techniques used for the detection and classification of different types of road anomalies.

The article "Edge AI-Based Automated Detection and Classification of Road Anomalies in VANET Using Deep Learning" was published in 2021. Journal: Comput Intell Neurosci.

In the future, the research can be broadened by adding more types of road anomalies and roads with multiple defects. Moreover, the automatic control of vehicle action based on anomaly type and prevention can be incorporated in an autonomous vehicle by using less complex deep learning models.

## Figures and Tables

**Figure 1:** Comparison of the road accident death rate in Asian countries.

**Figure 2:** Proposed mechanism for road anomaly detection in VANET.

**Figure 3:** Steps in proposed methodology for automated detection and classification of road anomalies.

**Figure 4:** General architecture of ResNet-18 for road anomalies classification.

**Figure 5:** General architecture of VGG-11 for road anomalies classification.

**Figure 6:** Training and validation loss of ResNet-18.

**Figure 7:** Confusion matrix for ResNet-18.

**Figure 8:** Training and validation loss of VGG-11.

**Figure 9:** Confusion matrix for VGG-11.

**Figure 10:** Comparison of ResNet-18 and VGG-11 accuracy for road anomalies classification.

**Figure 11:** Comparison of different techniques for pothole detection.

**Figure 12:** Comparison of different techniques for road bump detection.

**Figure 13:** Comparison of different techniques for crack detection.

**Table 1:** Distribution of road anomalies' dataset.

Road anomaly	Before augmentation	After augmentation
Pothole	263	1237
Bump	118	1008
Crack	118	1170
No anomaly	130	1113

**Table 2:** Input parameters for models' training.

S. no.	Parameter	Value
1	Image size	224
2	Batch size	64
3	Random seed	42
4	Num of epochs	10
5	Learning rate	0.001

**Table 3:** Result of evaluation parameters for ResNet-18.

S. no.	Road anomaly	Prc (%)	Rec (%)	Acc (%)	Fs (%)
1	Bump	100	99.70	99.92	99.84
2	Crack	100	100	100	100
3	No anomaly	99.38	100	99.85	99.68
4	Pothole	100	99.73	99.92	99.86

**Table 4:** Result of evaluation parameters for VGG-11.

S. no	Road anomaly	Prc (%)	Rec (%)	Acc (%)	Fs (%)
1	Bump	100	100	100	100
2	Crack	99.41	100	99.85	99.70
3	No anomaly	100	100	100	100
4	Pothole	100	99.43	99.85	99.71

**Table 5:** Comparison of proposed techniques with previous vision-based techniques.

Reference	Dataset	Anomaly type	Technique	Prc (%)	Rec (%)	Acc (%)	Fs (%)
[22]	Private	Crack's area Road marking	CNN	90.81	74.40	NM	81.79
[23]	Private	Pothole	SV1 SV2 LM1 LM2	45.8 67.4 89.8 NM	45.8 51.2 92.8 NM	NM	NM
[25]	Private	Crack	FCN (VGGNet)	91.30	94.10	NM	92.10
[28]	Private	Speed bumps	Image filtering	NM	NM	90.00	NM
[26]	Private	Speed bumps	Morphological algorithm	NM	NM	84.50	NM
[30]	Private	Crack	Neural network (NN) Random forest (RF) Extremely-randomized trees (ERT) Support vector machine (SVM) Logistic regression (LR)	90 86 87 87 88	90 86 87 87 88	90 86 87 87 88	90 85 86 87 87
[32]	Public	Crack	FC-DenseNets	95.91	96.63	NM	96.27
[33]	Multiple datasets (Public + Private)	Pothole	CNN SVM	100 86.87	99.60 82.20	99.80 88.20	99.60 81.62
[34]	Public	Speed bumps	TensorFlow API	97.46	98.46	97.44	97.96
[35]	Public	Pothole	Yolov2	95.55	91.42	89.41	93.43
[38]	Public	Crack	CrackForest (one-class SVM)	96.73	92.53	NM	94.58
[39]	Private	Crack	CNN	86.96	92.51	NM	89.65
[42]	Public	Crack	MobileNetV2 EfficientNetB0 DenseNet201 InceptionV3	98.21 98.78 98.92 98.91	97.40 99.45 99.73 99.04	97.82 99.11 99.32 98.89	97.81 99.12 99.32 98.98
[47]	Public	Pothole	Canny edge detector	81.80	74.40	NM	NM
[48]	Private	Pothole	Morphological algorithm	80	73.30	73.50	NM
[49]	Public	Pothole	Thresholding Edge detection *K*-means clustering Fuzzy C-Means clustering	NM	64.04 67.34 87.18 71.39	80.60 90.19 82.47 82.46	NM
[53]	Private	Pothole	HOG and Naive Bayes	86.50	94.10	90.00	NM
[79]	Public	Pothole Bump Normal	YOLO based on ResNet-50	NM	NM	NM	NM
[29]	Public	Pothole	YOLOv3 SSD HOG Faster-RCNN	NM	NM	82 80 27 74	NM
[37]	Public	Pothole	CNN	95.2	92	95	93.6
[50]	Private	Crack	CNN	57.7	67.2	70.7	62.1
Proposed	Multiple datasets (public)	Pothole Speed bumps Crack No anomaly	ResNet-18 VGG-11	99.85	99.85	99.92	99.85

The article "Edge AI-Based Automated Detection and Classification of Road Anomalies in VANET Using Deep Learning" was published in 2021. Journal: Comput Intell Neurosci.

## Data Availability

The datasets that have been used in the research are public datasets (https://www.kaggle.com/sachinpatel21/pothole-image-dataset, https://www.kaggle.com/virenbr11/pothole-and-plain-rode-images, https://data.mendeley.com/datasets/xt5bjdhy5g/1, and https://github.com/cuilimeng/CrackForest-dataset). The simulation data used to support the findings of this study are available from the corresponding author upon request.
